# Region Convolutional Neural Network for Brain Tumor Segmentation

**DOI:** 10.1155/2022/8335255

**Published:** 2022-09-10

**Authors:** R. Pitchai, K. Praveena, P. Murugeswari, Ashok Kumar, M. K. Mariam Bee, Nouf M. Alyami, R. S. Sundaram, B. Srinivas, Lavanya Vadda, T. Prince

**Affiliations:** ^1^Department of Computer Science and Engineering, B V Raju Institute of Technology, Narsapur 502313, Telangana, India; ^2^Department of Electronics and Communication Engineering, Sree Vidyanikethan Engineering College, Tirupati, Andhra Pradesh 517102, India; ^3^Department of Computer Science Engineering (Cyber Security), Karpagam College of Engineering, Coimbatore, Tamilnadu, India; ^4^Department of Computer Science, Banasthali Vidyapith, Aliyabad 304022, Rajasthan, India; ^5^Department of Electronics and Communication Engineering, Saveetha School of Engineering Saveetha Institute of Medical and Technical Sciences, Chennai 602105, Tamil Nadu, India; ^6^Department of Zoology, College of Science, King Saud University, P. O. Box 2455, Riyadh 11451, Saudi Arabia; ^7^Department of Health Sciences, University of Texas, Austin, TX, USA; ^8^Department of Electronics and Communication Engineering, Maharaj Vijayaram Gajapathi Raj College of Engineering (A), Vizianagaram 535005, Andhra Pradesh, India; ^9^Department of Computer Science, Woldia Institute of Technology, Woldia University, North Wollo, Ethiopia

## Abstract

Gliomas are often difficult to find and distinguish using typical manual segmentation approaches because of their vast range of changes in size, shape, and appearance. Furthermore, the manual annotation of cancer tissue segmentation under the close supervision of a human professional is both time-consuming and exhausting to perform. It will be easier and faster in the future to get accurate and quick diagnoses and treatments thanks to automated segmentation and survival rate prediction models that can be used now. In this article, a segmentation model is designed using RCNN that enables automatic prognosis on brain tumors using MRI. The study adopts a U-Net encoder for capturing the features during the training of the model. The feature extraction extracts geometric features for the estimation of tumor size. It is seen that the shape, location, and size of a tumor are significant factors in the estimation of prognosis. The experimental methods are conducted to test the efficacy of the model, and the results of the simulation show that the proposed method achieves a reduced error rate with increased accuracy than other methods.

## 1. Introduction

Patients suffering from brain tumors are particularly sensitive to the debilitating effects of the disease [1], which can be fatal. There are two types of brain tumors: primary tumors that begin and secondary tumors that begin in other body parts and spread to the brain as a result of the spread of malignant cells. Primary tumors are those that begin in the brain cells and spread to other parts of the body. Primary tumors such as gliomas are among the most frequent types of tumors [2–4]. However, glial cells in the brain are not alone in being afflicted; the disease has also extended to the tissue around them. In comparison, astrocytoma, which is a low-grade glioma (LGG) that grows more slowly, has a longer overall survival time. There are a lot of ways to treat cancer, including radiotherapy and chemotherapy that can either kill or slow the growth of tumor cells that cannot be removed through surgery. Consequently, for many brain tumors, neurosurgery remains the first, and in some cases, the only therapy option is available to the patient. In addition to the difficulty associated with the complexity of the brain anatomy, modern surgical approaches for treating brain tumors are fraught with danger. For neurosurgeons, visual inspection alone is insufficient for distinguishing tumor tissue from normal brain parenchyma [5, 6].

Most brain tumors are found and treated during surgery with magnetic resonance imaging (MRI), which is a noninvasive imaging technology based on magnetic resonance. MRI also has the benefit of providing detailed images of vascularity and cellularity of the brain tumor as well as the blood-brain barrier thanks to the use of multimodal protocols, which may be performed simultaneously. These images can be used by neurosurgeons to aid in the diagnosis and treatment of their patients. In order to analyze these data during neurosurgery, it is vital to have a correct representation of the lesion shape that is distinct from healthy brain regions [7]. The manual segmentation of brain tumor is required in order to accurately determine the position and nature of the tumor. This is done by a team of medical professionals. Aside from that, the method of lesion localization is time-consuming and significantly relies on the physician's previous knowledge, skill, and split-second decisions. Computer-based segmentation procedures, on the other hand, are a viable alternative to manual segmentation methods because they cut down on the amount of time and effort that surgeons need to spend on diagnostic or assessment operations while still giving accurate and trustworthy results [8]. Machine learning algorithms for identifying normal and sick brain tissue from magnetic resonance imaging (MRI) images have been developed in the past [9, 10].

The selection of parts that will allow this operation to be completely automated will necessitate the use of computer engineering and medical expertise. In order to avoid this, traditional methods are highly dependent on the unique application and are therefore not very generalizable. Due to their variability in shape, size, and position, malignant areas are difficult to recognize and can only be described by changes in the intensity of the cells in comparison to healthy cells. As a result, it is challenging to develop fully automated brain tumor treatment processes. It should be noted that there are two main drawbacks to this approach: Because the training patches are far larger in size than the training samples, it takes significantly more computation cycles to run them. A second aspect that influences segmentation accuracy is the size of the patch that should be applied. By using augmented data, networks can deliver effective segmentation even with only a few training images, which is a remarkable achievement in machine learning. Tiling is also capable of using high-resolution images while still utilizing a small amount of GPU RAM for training purposes.

Different methods are being followed in diagnosing cancerous tumors. In particular, the development of machine learning methods helps to improve it further. The importance of these methods was analyzed in terms of the size and shape of the cancerous tumors that are malignant. Thus, the calculation of its exact location and treatment methods gave delayed results. Analyses are currently being carried out to rectify this, and the boundaries have been defined based on its results and its results have been rendered correctly. In this article, a segmentation model is designed using RCNN that enables automatic prognosis on brain tumors using MRI. The study adopts a U-Net encoder for capturing the features during the training of the model. The feature extraction extracts geometric features for the estimation of tumor size. It is seen that the shape, location, and size of a tumor are significant factors in the estimation of prognosis.

## 2. Related Works

It was also the focus of two recent studies, one in [10] and the other in [11], which summarized standard brain tumor segmentation approaches. Both of them lacked a technical analysis and description of deep learning-based segmentation methods, which were necessary for their respective fields. As revealed by an early analysis of currently available approaches [12], machine learning models and characteristics are frequently employed in the segmentation of brain tumors.

An investigation of magnetic resonance imaging (MRI)-based brain tumor segmentation was reported in [13]. According to the results, deep learning-based methodologies are not included in this survey. The authors in [14] looked at the technical aspects and consequences of different types of data augmentation methods. We focused on the technical aspects of deep learning-based approaches for brain tumor segmentation. An increasing number of representative polls on the same issues have been conducted in recent years. Refs. [15–20] provided a summary of novel medical image analysis applications based on deep learning algorithms that have been developed. This study gives an overview of medical image analysis studies that were done, as well as some new, cutting-edge algorithms that use deep learning to separate brain tumors from healthy parts of the brain.

The authors in [21] conducted a review of the use of deep convolutional neural networks for brain image analysis. In this article, deep convolutional neural networks are only briefly explored. It was not covered in this study whether segmentation under imbalanced situations and multi-modality learning is possible. The authors in [16–18] did a survey of deep learning for the purpose of brain MRI segmentation. This work [19] published a survey on deep learning for healthcare objectives that was recently published. Healthcare applications are being improved through the use of computer vision, natural language processing, reinforcement-learning, and generalized methodologies, among other techniques. The goal of a survey released very recently [22] was to discover the consequences of object detection and semantic segmentation for machine learning.

When it comes to the segmentation of brain tumors, there are several questions that remain unresolved. The purpose of brain tissue segmentation, also known as anatomical brain segmentation, is to assign a distinct brain tissue class to each individual unit in order to better understand the brain. They must assume that the brain imaging does not reveal any tumor tissue or other abnormalities in order to finish their assignment. Aiming for the separation of the white matter lesion from the surrounding brain tissue is what white matter lesion segmentation is all about. The white matter lesion does not have subregions like tumor cores, which means that binary classification methods cannot be used to segment the lesion in its current task. The purpose of tumor identification is to identify any abnormal growths or lesions in the body and to provide information on the tissue predicted classification, which is accomplished through biopsy.

The detection result is normally represented by the bounding box, and the classification result is typically represented by the labels [23–25]. There are some approaches to brain tumor segmentation that just provide the single label segmentation mask or the tumor core center point without generating subregion segmentation results, and this is something that should be brought to your attention as a result. This article describes tumor segmentation using subregional semantic segmentation, which is based on subregional semantic segmentation. Signs of disorders such as high- and low-grade gliomas, moderate cognitive impairment, Alzheimer's disease, and schizophrenia are looked for on brain scans. Aside from identifying tumor patterns and activities, survival prediction [26] may also forecast survival rates [27] by identifying patterns and activities in tumors. The disease categorization and survival prediction can be classified as downstream jobs based on the results of tumor segmentation, and both tasks can be classified as downstream tasks.

## 3. Proposed Method

The RCNN [20] architecture includes a 3D attention module that is integrated with decoder blocks. In order to improve segmentation prediction, a 3D attention model with decoder blocks has been presented. This proposed attention module includes three components: a skip connection and channel, as well as spatial attention. In contrast, combining features that are already interesting may make it difficult to learn new features when they are combined with other characteristics.  Figure 1 depicts the proposed design.

In the proposed method, the required data must first be obtained as input. Upscaling image blocks is done based on those inputs. The data in that upscaling system are subdivided into different quality groups, and the classification of the data is further enhanced as the results of the classifications are further presented.

### 3.1. Image Upscaling

In semantic segmentation, the effective use of both semantic and geographical information is important to the neural network's capacity to perform successfully. As a result, the decoder must recover the spatial information in order to produce a segmented map using the spatial information recovered by the decoder.

A few adjustments were made to the U-Net decoder in order to generate even better segmentation results in the final analysis. A BN is found between ReLU and the convolutional layer, allowing the different layers to learn independently of one another, resulting in shorter training durations. Finally, the outputs are fed into a SoftMax layer output, which provides a list of probability distributions based on the network output logic.

### 3.2. Classification

There are three layers in each step of standard CNNs: a convolution layer, a feature pooling layer, and a fully connected layer (FC).

The feature maps from the previous layers are convolved with learnable kernels *k*_*ij*_^*l*^ at the convolution layer, and a bias parameter (*b*_*j*_) is also included in the process. It is then passed via an activation function *f* (•), which produces an output feature map, which can subsequently be used to train the system. The following is a concise summary of the procedure as in,

(1) $$\begin{array}{c} X_{j}^{l}=f\left(\sum_{i\in M_{j}}X_{i}^{l-1}k_{ij}^{l}+b_{j}^{l}\right), \end{array}$$

where *M*_*j*_ is input map selection.

### 3.3. Feature Pooling Layer

This layer is responsible for handling a single feature map. There are a lot of subsampling layers, and this particular one is referred to as a down-sampling layer in the industry. This results in the same number of input and output maps as before, but the output maps are smaller in size than the input maps. A little modification in the features of the previous layer has no effect on the findings of the current layer. The following is a concise summary of the procedure as shown in the following equation:

(2) $$\begin{array}{c} X_{j}^{l}=\mathrm{down}\left(X_{i}^{l-1}\right), \end{array}$$

where down (·) is downsampling.

To make the input smaller, we use a technique called down-sampling, which is when neurons are put together from a small area of space.

### 3.4. Fully Connected (FC) Layers

After data have been processed by numerous convolutional and subsampling layers, the FC levels in the neural network conduct high-level reasoning on the input. The neurons in the FC layer are completely connected to the neurons in the preceding layer. After completing the matrix multiplication and bias offset, it is possible to compute their activation states. As illustrated in Figure 2, the flowchart of a CNN demonstrates how it operates.

The first given image data are divided into small groups. These small groups consist of small data sets of their type and character. These groups are then paid in small sections based on the sequence codes for them. Then, it goes to pooling compilation. Here, the primary and final form pooling models are interconnected, and their designs are defined, re-convolved, and finally classified.

### 3.5. Train Phase

In order to train all of the network layer parameters during the training phase, the error backpropagation technique must be used, which is necessary because CNN is a somewhat deep neural network. As a result, there are only a limited number of remote sensing data sets accessible, making it very hard to manually categorize millions of images using training data. AlexNet is the pre-trained model that we utilize in our investigations, and it was trained on the ImageNet dataset. AlexNet was trained on the ImageNet dataset.

### 3.6. Test Phase

A test data set with 180 blocks that were cropped out of airport areas and 1132 different types of tumor was created in order to evaluate the proposed tumor identification system's effectiveness. A comparison of the precision and recall rates of the proposed RCNN approach with the standard BOVW method was carried out using test data collected for both methods. Our experiments on images of full airports, which are usually surrounded by a range of complex landscapes, were conducted in order to demonstrate the durability of the proposed tumor recognition system. An effective tumor detection system must be able to work well in many different types of environments.

We employed procedures such as selective search and other methods on an image that we had previously obtained in order to cut down the pool of prospective possibilities. Candidate regions are referred to as proposals in some circles, and they offer potential landing sites for airplanes. In our trials, we compared the effectiveness of these alternative tactics. The recall rate of sliding windows is always higher than that of other types of windows, but they are also the most time-consuming and have a large number of false positives. BING, the fastest algorithm, assigns a score to each tumor suggestion in order to indicate the level of confidence in the idea.

Therefore, we can only accept a certain number of entries, ranging from the most to the least favorable. Our research, on the other hand, has revealed that the final findings are never completely center-aligned with the object depicted in the final image. A score is assigned to each proposition by edge boxes, with the difference being that this number merely reflects how confident you are that the box contains a general item, rather than an airplane. There are a couple of genuine positives that are overlooked by edge-box results. This is done in order to avoid giving a low score to a legitimate tumor in a difficult position, as previously stated. In our tumor detecting system, we employ selective search as a means of generating propositions.

## 4. Results and Discussions

Python is used to implement proposed models in conjunction with the Tensor Flow backend. To put all of the suggested feature extraction networks to the test, we employed FLAIR MRI sequences with a resolution of 224 × 224. All networks are trained for 35 epochs with a batch size of 16, which is the maximum allowed. Following the feature extractor process, spatial dropout was used at a rate of 0.5 to further refine the results.

Regularization is a basic strategy for ensuring that neural networks generalize successfully without overfitting the training dataset, and it is used to achieve this goal. The learning rate of the Adam optimizer has been set to 0.00001% per second. Because of a data imbalance problem in the BraTS dataset, cancer pixels account for less than 2% of the dataset's total pixels, while healthy pixels account for 98% of the total pixels.

For this analysis, the FLAIR MRI data from the BraTS 2019 challenge was used as the basis. The use of fluorescence in situ angiography (FLAIR) for glioma imaging is becoming increasingly essential because of a growing trend to eliminate FLAIR-positive regions from glioma tumors. The BraTS dataset contains preoperative magnetic resonance imaging (MRI) images of 336 glioma patients from a variety of institutions.

Depending on the patient needs, four different types of scans are performed: a native *T*1-weighted scan, a post contrasted *T*1-weighted scan, a *T*2-weighted scan, and, for those who are eligible, a *T*2-FLAIR scan. Nineteen universities contributed MRI data from a range of clinical regimens and scanners. Expert neuroradiologists manually separated the data from 1 to 4 using the same annotation process that they used to segment the data from 1 to 4. In the next step, the MRI scans are interpolated to the same resolution of 1mm^3^ and resampled.

It is possible that bias field noise, which may be defined as undesirable artifacts that occur during the image collection process, will affect the training images since they come from a range of sources, methodologies, and institutions, and will affect the training images. In order to eliminate these effects, the revised *N*3 bias correction tool is utilized to perform image-wise normalization and bias correction on each individual image. After that, the data for each FLAIR MRI slice are normalized by subtracting the mean and dividing it by the standard deviation of the slice data, and the data for each slice are then normalized again.

When training large neural networks with a limited amount of training data, it is important to exercise caution in order to avoid the problem of overfitting. Many ways can be used to improve the performance of a model, such as adding new artificial training data to existing training data in order to make the model more general and improve its performance as shown in Figure 3–Figure 7.

As part of our effort to validate the efficacy and durability of the proposed detection system, we measured the performance of the system using the test data provided. For performance evaluation, more than 60% of the tumor can be detected in the detection window that has been set aside. The following equations are the definitions for precision and recall rates:

(3) $$\begin{array}{c} \text{Precision}=\left(\frac{\text{TP}}{\text{TP}+\text{FP}}\right), \end{array}$$

(4) $$\begin{array}{c} \text{Recall rate}=\left(\frac{\text{TP}}{\text{TP}+\text{TN}}\right). \end{array}$$

Data augmentation processes, such as horizontal and vertical flips, rotations, scalings, and shearings, are employed in this study to improve the quality of the data as it is being collected and processed. Simply using these types of methodologies does not provide enough data for immune training, which is why more complex methods such as elastic distortion, which corresponds to uncontrolled noise in MRI sensors, are being added. In this method, deformation intensity is controlled by the elasticity coefficient *σ* and the multiplying factor *α* of displacement fields, which are both positive numbers.

When compared to the validation set, the deep learning architectures presented were able to accurately detect cancer regions with mean DSC scores that ranged from 0.8009 to 0.8439. The mean dice score of the expert annotation for the entire tumor core, on the other hand, was roughly 0.85. This means that completely automated deep learning models could be used to separate brain tumors, even though the statistical analysis of their results is almost the same.

Despite the fact that the Xception encoder achieved a higher sensitivity score of 0.856 than the original U-Net model, it achieved a poorer specificity score of the same value. In this study, it was discovered that point-based procedures are insufficient for evaluating the accuracy of brain tumor segmentation algorithms. As a result, high-definition measurements were used to figure out which deep encoder had the best accuracy and performance out of the other ones that were tested. Figure 3 depicts the accuracy.

The proposed architectures are based on data from the validation set. In each figure, there are two rows, one displaying FLAIR images in greyscale mode and the other displaying manual ground truth segmentations created manually.  Figure 4 shows the precision.  Figure 5 depicts the recall.  Figure 6 depicts the F-measure, and Figure 7 shows the MAPE. The results of several automatic segmentation techniques are displayed in the following rows, which are arranged in descending order. Recommended encoders can make borders for tumors that are very similar to those that are manually labeled, even if the lesion shape, volume, and texture change a lot.

Various methods of diagnosing cancerous tumors in general have come into practice. Its use is determined by its accuracy and its special features. In that sense, the proposed algorithm is considered to be better than the given algorithms. Its results make it clear that its accuracy and cancer detection methods are excellent. Furthermore, its boundaries are defined and analyses are performed correctly so that the size and shape of the cancerous tumor can be accurately calculated and its location accurately calculated. Thus, the doctor can prescribe the right treatment to the patient depending on where it is located.

## 5. Conclusions

In this article, a segmentation model is designed using RCNN that enables automatic prognosis on brain tumors using MRI. The study adopts a U-Net encoder for capturing the features during the training of the model. The identification of objects in optical remote sensing images has become a study focus in recent years. Advances in object detection have been made possible thanks to the use of deep learning, particularly RCNN. Numerous improvements to RCNN are presented in optical remote sensing. As a result, dilated convolutions are used to get better results when we look at optical remote sensing images of dense things. The feature extraction extracts geometric features for the estimation of tumor size. It is seen that the shape, location, and size of tumor are significant factors in the estimation of prognosis. The exact location of the tumor was classified, and the type of cancer predictions are planned to be implemented in the next phase. It is very useful for doctors to identify the cancer types and the treatment methods. This will also be helpful for the patients to know about the stage of cancer and follow the doctor's proper medical treatments.

## Figures and Tables

**Figure 1:** Proposed design.

**Figure 2:** Flowchart of RCNN.

**Figure 3:** Accuracy.

**Figure 4:** Precision.

**Figure 5:** Recall.

**Figure 6:** *F*-measure.

**Figure 7:** MAPE.

## Data Availability

The data used to support the findings of this study are included within the article. Further data or information is available from the corresponding author upon request.
